The article "Is Femoral Nerve Block Superior to Fascia Iliac Block in Hip Surgery? Meta-Analysis of Randomized Controlled Trials" was published in 2022. Journal: Biomed Res Int.

# Is Femoral Nerve Block Superior to Fascia Iliac Block in Hip Surgery? Meta-Analysis of Randomized Controlled Trials

**DOI:** 10.1155/2022/4840501

**Published:** 2022-05-19

**Authors:** Xiao-dan Li, Chao Han, Wen-li Yu

**Affiliations:** ^1^Department of Anesthesiology, Tianjin First Central Hospital, No. 24 Fukang Road, Nankai District, Tianjin 300192, China; ^2^Department of Orthopedics, Tianjin Hospital, No. 406 Jiefang South Road, Hexi District, Tianjin 300211, China

## Abstract

**Background:**

Femoral nerve block (FNB) and fascia iliac compartment block (FICB) are alternative methods of pain relief during hip surgery. Nevertheless, the effectiveness and safety of FNB compared with FICB are yet to be fully determined.

**Methods:**

Electronic databases were systematically searched. Only randomized controlled trials (RCTs) on hip surgery were included. Postoperatively, the pain scores at different time points, narcotic requirements in 24 h, mean arterial pressure, spinal anesthesia (SA) time, patient satisfaction, and adverse effect rates between the two groups were extracted throughout the study.

**Results:**

Fourteen RCTs including 1179 patients were included. Compared to the FICB, FNB decreased the VAS scores postoperatively at 24 h at rest (*P* < 0.05) and the incidence rate of some side effects (nausea, vomiting, and sedation) (*P* < 0.05). However, compared to the FICB, no significant difference was found in the FNB regarding the VAS scores postoperatively at any of the other time points (2 min, 20 min, 2 h, 24 h at movement, 48 h at rest, and 48 h at movement). Patients in both groups had similar narcotic needs after 24 h, mean arterial pressure, SA time, and patient satisfaction (*P* > 0.05).

**Conclusions:**

FNB has more advantages in reducing VAS scores postoperatively at 24 h at rest and the odds of some adverse effects. A better quality RCT is needed to properly compare FNB with FICB.

## 1. Introduction

Hip surgery-related pain occurs often, and it is commonly treated poorly because of the patient's advanced age, comorbidities, and increased sensitivity to the side effects of analgesics [1]. Although it may be helpful to improve the surgical techniques and the perioperative period management, many patients still suffer from tremendous pain after hip surgery. A number of complications, such as lower limb deep venous thrombosis and bedsore, can arise as a consequence of postoperative procedures, causing hospitalization and increased medical costs [2]. It is crucial in clinical practice that the appropriate management is adopted to manage postoperative pain under such circumstances [3].

The postoperative pain score, the dose of the analgesic required, the mean arterial pressure, and the time during which anesthesia was administered, as well as the incidence of anesthesia-related adverse effects, were often applied to evaluate the effect of anesthesia [4–6]. The patient may experience intractable postoperative pain if inappropriate methods of anesthesia were used [7]. The use of peripheral nerve blocks as a pain management strategy has been recommended following hip surgery due to the adverse effects of opioid analgesics [3]. Under such circumstances, a femoral nerve block (FNB) and fascia iliac block (FICB) have been proven to result in a lower rate of complications and better pain control in the elderly [8].

Several studies have been conducted in the past decades on the effects of FNBs and FICBs, perioperatively [9–11]. While some conclusions have been made, whether FNB is equivalent to FICB in pain relief for hip surgery has rarely been studied through meta-analyses. The aim of this study was to compare the effects of FNB and FIB on the reduction of pain and side effects in randomized controlled trials (RCTs).

## 2. Methods

The PRISMA statement [12] was followed for this meta-analysis. Since this was a report on the published literature, no ethical approval was required. A comprehensive list of all literature identified by electronic searches, including MEDLINE (1966–present), EMBASE (1966–present), and Cochrane Central Register of Controlled Trials. To increase the search accuracy, the following keywords were combined with MeSH terms: “pain management, postoperative pain, hip surgery, hip fractures, femoral fractures, hip replacement, hip arthroscopy, FNBs, and fascia iliac compartment blocks.” Only RCTs in humans have been conducted up to August 2021. PRISMA Flow Diagram (Figure 1) is seen below.

### 2.1. Inclusion Criteria

Literature was considered eligible for inclusion if it satisfied the following requirements: types of studies: RCTs and reports in English; population: hip surgery patients; types of interventions: FNB and FICB; and types of outcomes: a minimum of one of the following items was reported: total morphine consumption, visual analog scale (VAS) score, spinal anesthesia (SA) time (as defined as time from the start of positioning to drug injection completion), mean arterial pressure, patient satisfaction, and side effects.

### 2.2. Exclusion Criteria

Patients with neoplasms, severe osteoporosis, infections, metal sensitivity, and mental diseases were excluded from this study.

### 2.3. Selection Criteria

Two independent reviewers conducted the eligibility assessments. A dispute between reviewers was resolved through discussion; if there was no consensus, the third reviewer made the final decision. The RCTs were evaluated using funnel plots to determine the risk of bias according to the Cochrane Collaboration tool [13].

### 2.4. Data Extraction

A pooled analysis of data from the included studies was independently performed by two authors (Xiao-dan Li and Chao Han). Data from the following sources were extracted and analyzed: first author's name, anesthesia type, types and methods of narcotics, pain assessment methods, and adverse reactions are all listed along with the publication year. Data that could not be clarified or were incomplete were contacted by the authors to retrieve missing information.

### 2.5. Statistical Analysis

The pooled data were analyzed using RevMan5.3 (Cochrane Collaboration, Oxford, UK). *P* and *I*^2^ values were calculated using the chi-square test to measure heterogeneity. *P* > 0.10 and *I*^2^ < 50% were defined as having no significant heterogeneity, and an analysis of data using fixed-effects models was then conducted. In the case of significant heterogeneity, an effect model with random effects was applied. The mean difference (MD) and 95% confidence intervals (CIs) of continuous outcomes, such as VAS scores and narcotic consumption, were pooled to make reports. The relative risks were calculated with 95% CIs for dichotomous data, such as vomiting and nausea. Statistical significance was set at *P* < 0.05.

## 3. Results

### 3.1. Literature Search

An electronic search yielded 861 potential records, including 229 duplicate articles. Six hundred and eighty-eight articles were identified as irrelevant by the titles and excerpts, leaving fourteen studies that eventually met the eligibility requirements [4–6, 14–24]. The 14 RCTs enrolled 590 patients on the FNB group and 588 patients on the FICB group. Publications took place between 2011 and 2020.

### 3.2. Study Characteristics

As shown in Table 1, the included studies were characterized by the following key characteristics: all available literature consists of relatively small sample sizes, ranging from 10 to 85 patients. Preoperatively nerve block was applied in 13 studies [4–6, 14–18, 20–24], and postoperative nerve block was used in 1 study [19]. 5 studies [6, 16, 20, 22, 23] employed the general anesthesia, 4 studies [4, 5, 14, 19] used regional anesthesia, and 5 studies [15, 17, 18, 21, 24] did not mention the detailed method of anesthesia. Fentanyl was used for standard general anesthesia. Two groups of statistical characteristics were analyzed.

### 3.3. Assessment of Risk Bias

All included RCTs were evaluated for bias using the Cochrane Collaboration tool.  Figure 2 shows a quality assessment of the methodology. All included studies had a low risk of bias.

## 4. Outcomes for Meta-Analysis

### 4.1. Postoperative VAS Scores at Different Time Points

Details regarding postoperative VAS at different time points (2 min, 20 min, 2 h, 24 h at rest, 24 h at movement, 48 h at rest, and 48 h at movement) were available in 12 trials [4–6, 15–22, 24]. Significant heterogeneity was found (*P* < 0.05) in the VAS at 2 h, VAS at 24 h at rest, and VAS at 24 h at movement. The results showed that compared to the FICB, the FNB could decrease the VAS postoperatively at 24 h at rest (MD = −0.46, 95% CI: -0.86 to -0.06, *P* = 0.03). There was no significant difference in the FNB compared with the FICB at the rest time points postoperatively (2 min, 20 min, 2 h, 24 h at movement, 48 h at rest, and 48 h at movement) (MD = 0.08, 95% CI: -0.12 to 0.28, *P* = 0.46) (MD = −0.24, 95% CI: -0.54 to 0.07, *P* = 0.13) (MD = −0.23, 95% CI: -1.21 to 0.75, *P* = 0.65) (MD = −0.16, 95% CI: -1.04 to 0.72, *P* = 0.72) (MD = −0.10, 95% CI: -0.30 to 0.11, *P* = 0.36) (MD = −0.25, 95% CI: -0.60 to 0.11, *P* = 0.17Figure 3).

### 4.2. Narcotic Requirements at 24 h

There were four trials that reported details of narcotic consumption [18, 20, 22, 23]. In the meta-analysis, a significant heterogeneity was found (*P* < 0.05), and no significant differences were shown in the FNB groups compared with the FICB group in reducing narcotic consumption at 24 h (MD = 0.45, 95% CI: −0.30 to 1.20, *P* = 0.24Figure 4).

### 4.3. SA Time

Three trials evaluated the SA time in the two groups [4, 5, 14]. Significant heterogeneity was found (*P* < 0.05); the random model was used. Compared with the FIBC group, no significant difference in SA time was found in the FNB group (MD = −9.13, 95% CI: -61.28 to 43.03, *P* = 0.73; Figure 5).

### 4.4. Mean Arterial Pressure (mmHg)

Two trials compared the mean arterial pressure in two groups [6, 17]. Heterogeneity did not appear to be significant (*P* > 0.05), a fixed model was made. Compared with the FIBC group, no significant difference in the mean arterial pressure was found in the FNB group (MD = −1.11, 95% CI: -5.00 to 2.79, *P* = 0.58; Figure 6).

### 4.5. Patient Satisfaction

Details regarding patient satisfaction were available in four trials [5, 14, 16, 22]. No significant heterogeneity was found (*P* > 0.05), and a fixed model was performed. No significant difference was found between the groups (relative rate 0.99, 95% CI: 0.84 to 1.17, *P* > 0.05; Figure 7).

### 4.6. Adverse Effects (Nausea, Vomiting, and Sedation)

Three studies reported nausea, vomiting, and sedation statistics [4, 6, 17]. Significant heterogeneity was not found in the included studies; therefore, a fixed-model was used (*P* > 0.05). Compared with FICB, FNB could significantly decrease the incidence of nausea, vomiting, and sedation, respectively (relative rate 0.30, 95% CI: 0.12 to 0.79, *P* < 0.05) (relative rate 0.13, 95% CI: 0.02 to 0.71, *P* < 0.05) (relative rate 0.40, 95% CI: 0.18 to 0.88, *P* < 0.05; Figure 8).

## 5. Results of Reporting Bias

A funnel plot was used to evaluate reporting bias. The diagram (Figure 9) demonstrates a low risk of publication bias. Egger's (*P* = 0.19) and Bagger's tests (*P* = 0.161) were also used to measure the level of reporting bias. In our meta-analysis, no reporting bias was observed.

## 6. Discussion

By analyzing the pooled data, we aimed to evaluate the relevant literature effectively and provide a better understanding of the usefulness of FNB and FICB for hip surgery. Our overall results show that FNB has more advantages in reducing VAS scores postoperatively at 24 h at rest and the incidence rate of nausea, vomiting, and sedation, respectively. The low incidence of those side effects can not only effectively improve patient satisfaction but also help patients recover faster after surgery [25]. Our meta-analysis confirms previous studies reporting decreased postoperative side effects associated with FNB [3, 26, 27].

The VAS score can serve as a good indicator of the extent of postoperative pain relief following hip surgery. Our work revealed that both FNB and FICB could alleviate pain, and FNB showed stronger analgesic ability at 24 h at rest postoperatively. However, no significant differences were observed at the other time points (2 min, 20 min, 2 h, 24 h at movement, 48 h at rest, and 48 h at movement). A wide range of factors may contribute to this, such as the severity of the fracture, type of surgery, and complications of the patient. Postoperatively, only patients in good condition can undergo early rehabilitation. As a result of better pain management, therapy costs and time can be reduced, which has a profound effect on patient recovery [28].

Decreasing opioid usage is important for better patient recovery. To assess the safety of FNB and FICB in the clinic, opioid requirements at 24 h were often employed. The UK National Institute of Health and Care Excellence recommends peripheral nerve block as an opioid-saving strategy. Both FNB and FIB were able to substantially minimize opioid consumption in this part, and no significant differences were observed between them. As with previous studies, our findings are in line with those of others [29, 30].

SA time, mean arterial pressure, and patient satisfaction were the common indices in the postoperative period to compare the efficacy between FNB and FICB. As shown in Figures 5–7, FNB and FICB shared a similar ability to handle these issues. Better pain relief, shorter time for SA, and more stable mean artery pressure with FNB and FICB are well reflected in the satisfaction of the patient perioperatively. The present study is comparable to previous studies that showed that FNB or FICB was more effective in decreasing pain, shortening the time to perform SA, and increasing patient satisfaction [30, 31].

To our knowledge, this meta-analysis is the first to compare the differences between FNB and FICB in the treatment of hip surgery. Since observational and retrospective studies have their limitations, all included studies were RCTs. Nevertheless, the heterogeneity of these studies may be determined by the study design and analysis methods. One limitation of the meta-analysis is that some variables such as hip surgery type, length of operation, and complications may also have a significant impact on the degree of pain, different types of anesthetics and dosages were used, and the levels varied between 15 mL and 50 mL for the various trials. Therefore, it is necessary to further investigate the optimal use of FNB and FICB.

Finally, because almost all the studies included in the review were conducted by anesthetists, several important details such as operative procedures, types, and methods of the operation were not reported. In future studies, it is necessary to take these factors into account, because this information may often be crucial for surgeons and directly affect the degree of postoperative pain.

## 7. Conclusion

According to this meta-analysis of RCTs, FNB helped to reduce VAS at 24 h at rest postoperatively and side effects (nausea, vomiting, and sedation) compared to the FICB. No significant difference was found in VAS at the rest of the time points, a narcotic requirement in 24 h, SA time, mean artery pressure, and patient satisfaction between FNB and FICB. More high-quality RCTs are necessary for proper comparisons of the efficacy and safety of FNB and FICB.

## Figures and Tables

**Figure 1:** The PRISMA flow diagram of included studies.

**Figure 2:** The bias risk of all trials.

**Figure 3:** Forest plot of postoperative VAS at different time points (2 min, 20 min, 2 h, 24 h at rest, 24 h at movement, 48 h at rest, and 48 h at movement).

**Figure 4:** Forest plot of narcotic consumption at 24 h between the two groups.

**Figure 5:** Forest plot of spinal anesthesia time between the two groups.

**Figure 6:** Forest plot of the mean arterial pressure (mmHg) between the two groups.

**Figure 7:** Forest plot of satisfaction for treatment between the two groups.

**Figure 8:** Forest plot of adverse effects (nausea, vomiting, and sedation) between the two groups.

**Figure 9:** Funnel plot of VAS score at 2  h.

**Table 1:** Characteristics of the included studies.

Clinical trials	FNB/FICB						Anesthesia	Dose of FNB	Dose of FICB	Reference type	Location
	Cases	Age (mean)	Gender (% male)	ASA grade (cases)							
				I	II	III					
Bantie 2020	24/24	37.7/34.2	21/22	20/19	4/5	N/A	Spinal anesthesia	30 mL of 1% lidocaine with adrenaline solution	30 mL of 1% lidocaine with adrenaline solution	RCT	Ethiopia
Blackwell 2021	37/21	N/A	N/A	N/A	N/A	N/A	General anesthesia	40 mL 0.5% ropivacaine	40 mL 0.5% ropivacaine	RCT	U.S.A.
Cooper 2019	48/52	84/80	12/16	N/A	N/A	N/A	Not mentioned	20 mL of 0.5% levobupivacaine and 20 mL 0.9% saline	20 mL of 0.5% levobupivacaine and 20 mL 0.9% saline	RCT	Australia
Deniz 2014	20/20	67.8/59.1	11/8	9/12	9/6	2/2	General anesthesia	2% prilocaine and 30 mL 0.25% bupivacaine	2% prilocaine and 30 mL 0.25% bupivacaine	RCT	Turkey
Ghimire 2015	15/15	55/54.4	7/10	5/6	10/9	N/A	Spinal anesthesia	15 mL 1.5% lignocaine with adrenaline	30 mL 1.5% lignocaine with adrenaline	RCT	Nepal
Liang 2020	23/23	74.3/73.9	6/7	N/A	17/17	6/6	Spinal anesthesia	15 mL 0.5% ropivacaine	40 mL 0.5% ropivacaine	RCT	China
Möller 2011	40/40	64/62	23/21	N/A	N/A	N/A	General anesthesia	50 mL prilocaine	50 mL prilocaine	RCT	Germany
Newman 2013	51/56	83/82	12/16	N/A	N/A	N/A	Not mentioned	0.5% levobupivacaine (30 mL for >70 kg; 25 mL for 50–70 kg; 20 mL for <50 kg)	0.5% levobupivacaine (30 mL for >70 kg; 25 mL for 50–70 kg; 20 mL for <50 kg)	RCT	UK

## Abbreviations

FNB: Femoral nerve block
FICB: Fascia iliac compartment blocks
VAS: Visual analog scale scores
SA: Spinal anesthesia
PRISMA: Preferred Reporting Items for Systematic Reviews and Meta-analyses
RCTs: Randomized controlled trials
MD: Mean difference
CI: Confidence intervals
RR: Relative risk.
